# B/S-Based Construction of a Big Data Logistics Platform

This article has been retracted.

**DOI:** 10.1155/2022/6873062

**Published:** 2022-07-13

**Authors:** Li Zhang

**Affiliations:** School of Management, Xi'an University of Finance and Economics, Xi'an, Shaanxi, China

## Abstract

Due to the overwhelming characteristic of the Internet of Things, devices belonging to these networks are utilized in almost every domain of real life in order to improve the lifestyle of humans. However, these networks result in a huge amount of data related to different application domains, leading to another important research aspect, i.e., big data and cloud computing. Big data and cloud computing technologies in the logistics field have experienced initial contact, gradual penetration, and widespread application. Moreover, it supports traditional logistics to upgrade to smart logistics, aiming to achieve the fundamental requirements of today's logistics industry and reduce costs with enhanced efficiency. However, the big data and cloud computing wisdom logistics model still has many problems in the construction of logistics public information platforms, end coordination development, government platform construction, and so on, in order to solve the problems of low efficiency, high cost, and low service satisfaction of traditional logistics. In this article, we have designed a new big data-enabled logistics detection system that is based on B/S architecture, constructed a smart logistics model consisting of a supply subsystem, demand subsystem, and supervision subsystem, and finally realized the operation process of the smart logistics model based on big data cloud computing.

## 1. Introduction

Advancements in technology, especially device miniaturization, preferably in circuitry, have led to the development and realization of the Internet of Things in various application domains such as healthcare, logistics management information system (LMIS), and industry. It is important to note that IoT leads to the production or generation of massive databases for which sophisticated procedures are needed to analyze it for effective decision-making processes; for example, in LMIS, collected data could be used to improve proper and effective management of the logistics. LMIS is an integrated information management system (LMIS), which integrates information collection, integration, processing, storage, and service and is used to operate and manage logistics business [1–3]. The LMIS is an information management system that integrates information collection, integration, processing, storage, and service to operate and manage logistics business. The management and operation of modern logistics require logistics information management software to ensure every aspect of the work, especially the connection points of the different logistics links, for maintenance. The logistics information management system is the soul of modern logistics.

The utilization of information flow in conjunction with applicable information technology to build an integrated channel between various logistical operations and some type of integration process is the essence of a logistics information management system. Not only is information sharing the initial aim of the Internet, but it is also a basic element of logistics management system design. The link between the various parts of the system is made possible by the communication between the various types of information. This information could be shared through two different means of communication: either using traditional wired communication where applicable or wireless communication. Only through information sharing can the rational scheduling of resources be achieved. Therefore, the logistics activities must first ensure the smooth flow and sharing of information, and the whole process of activities must be based on fundamental information and only then can logistics activities be carried out in a normal and orderly manner. The use of modern information technology makes it possible for the use of modern information technology and enables various departments, manufacturers, and sales companies to be linked together in a network via the Internet. This facilitates the sharing of information between departments and even companies and the exchange and storage of information and information on resources between departments and companies at the fastest and lowest cost. This is also the most intuitive benefit of the logistics industry after network informatization.

The logistics information system makes it possible to coordinate the overall situation, gives full play to the advantages of logistics resources, and facilitates the rational organization of logistics activities. This not only saves costs but also greatly increases the efficiency of the work. The application of logistics information systems makes logistics activities break the restrictions of the traditional logistics activities in terms of geography and time zones, and the scope of logistics has developed from the same city to the whole country or even the whole world. The quality of service has also increased, and customers can now get the most up-to-date logistics information and feedback in a timely way. The enterprise's self-strict management is substantially aided by the newest logistical information and consumer feedback information. Accumulation and analysis of logistics information resources may also assist businesses in controlling surplus inventory, orienting production, and so forth. The use of logistics information systems allows the logistics sector to emerge from the “dark continent of the economy,” as well as making the logistics management of products transit status and cargo information more visible in logistics management, as well as information regarding commodities. It also enables supply chain management, improves information interaction and sharing, and facilitates business. Supply chain management has also been made possible by improved information interaction and sharing, which is conducive to business cooperation between companies through information network platforms and the full utilization of more available resources.

With the advent of information technology, the conventional pattern of the logistics industry has changed considerably, and now, improving the management efficiency of business systems has become the key to the whole logistics industry's development [4, 5]. Strengthening the management of logistics enterprises with information technology means using information technology to achieve immediate information sharing, improving the management efficiency of the entire enterprise, minimizing total costs, increasing customer satisfaction, and thus improving the enterprise's competitiveness [6, 7]. Additionally, it is essential to note that these techniques could improve the logistic services, especially those provided by the traditional systems. The development of information technology and automation tends to enhance the management efficiency of logistics enterprises. For large domestic logistics company enterprises, the level of information technology and automation gradually tends to mature, such as unmanned delivery machines and automatic sorting centers. However, there are still many small logistics enterprises whose information technology level is in a backward state, which not only reduces the customer experience index but also greatly reduces the efficiency of the staff. Therefore, it is urgent to improve the information management level of small- and medium-sized enterprises.

In this article, we have worked on developing an effective logistic information management system based on the core concepts of big data, which is usually collected through devices belonging to the Internet of Things and cloud platform. The proposed system not only resolves the aforementioned issues currently faced by the research community and industrial partners in the logistic domain, but at the same time, an efficient information management system is developed and realized. This system could be used with little modification in other application domains as well. Finally, devices belonging to the IoT networks are used only to collect data related to the problem domain.

We have arranged the remaining sections of the article as provided below.

Overall or complete construction of the proposed system and its various parts are explained in the subsequent section, where various parts of the system have been presented in detail. Then it is followed by the description of the business model used in this setup. The fuzzy model that is also used in the article to improve the design of the proposed system is described in the subsection. In Section 3, the implementation of the proposed logistics information system is reported along with a description of its various parts. Results of the proposed scheme with respect to various measures have been reported in Section 4. Finally, concluding remarks about the paper are provided.

## 2. The Overall Construction of the System

The design of this logistics information system contains four servers: a frontend web server, a backend web server, a customer relationship server, and an Oracle database server, as shown in Figure 1.

The frontend pages of the frontend user system are designed using the *j* Query framework, and the server side uses the Spring and Struts2 frameworks to receive frontend request data and process it. The backend management system is designed for internal management use, and the pages are simple and practical, so the frontend pages are designed using the Easy UI framework, which makes the page development much more efficient, thus saving more time for backend development. The server side is developed in layers using the MVC design pattern, using the SSH framework and integrating Spring Data JPA, a framework provided by Spring to simplify JPA development based on Hibernate, making the development of the DAO layer more efficient and thus allowing more focus on the implementation of business logic in the development process.

The customer relationship system is a secondary system that has no frontend page presentation and the server side is designed using the SSH framework, which is basically the same as the frontend system. Both the customer relationship system and the backend management system use the Oracle database to store data. Moreover, various queries are used to extract useful or required information from the pool of available data using the proposed approach. Since Oracle does not have an auto-grow type, the corresponding sequence needs to be maintained for data tables that require primary key auto-grow.

### 2.1. System Business Statement

A business process is a collection of logically related activities that span time and space to accomplish a goal or task of an enterprise. System operations have customer-oriented, cross-functional, cross-departmental, and cross-enterprise attributes. Analyzing the system's business process diagram is the most intuitive technique to analyze a business process. The business flow diagram clearly depicts the system's business logic and the connections between the various subsystems, assisting developers in identifying redundant system components, removing unreasonable system components in a timely manner, and optimizing and streamlining the system's operations.  Figure 2 shows the business flow diagram for this system development, which is a very visual depiction of the system's numerous business modules. The system's business logic may be grasped at a look. In China, there are several brands of logistics management software, most of which are aimed at small and medium-sized businesses. The problem is that the function is single, but this logistics management system is developed for medium and large enterprises, which can also be a more feature-rich enterprise information management platform.

As shown in Figure 2, users can register and log in via the Internet in the system's user management and become a customer of the company. Orders are placed by telephone or via the Internet, and the relevant departments, on receipt of the order, first check the availability of the goods in stock at the warehouse. The vehicle management involves the registration, viewing, and entry and exit of the vehicle, as well as the management of the vehicle according to the size, quantity, and weight of the goods. After the vehicle is dispatched, there is logistics management, also known as transport management, during which the information on the goods in transit is viewed and tracked to enhance the user experience. After the goods have been transported and signed, the financial management also accounts for the financial documents. Throughout the system process, the data generated are backed up for future data analysis and data recovery. As we know, recovery is one of the most vital features of any electronic system, and if an effective recovery process is available, then the customer would like to invest in those systems. In addition, the following is a diagram of the activities of several important operations during the development of the system. Because the system is relatively large, only the activity diagrams of the order management, warehouse management, and vehicle management parts of the system are given. The activity diagrams are used to clearly illustrate the workflow of the business implementation [8] and to facilitate understanding of the specific business activities of the system.

The order service shown in the order management activity diagram in Figure 3 is an important part of the system development process. When a customer registers in the system, they can place an order by accessing the system, and then an order is generated in the system. Order is generated in the system. If the customer does not complete the payment within the specified time or if the customer cancels the order, the order activity will be canceled accordingly. After the customer has successfully paid, the order task will be assigned to the warehouse for the ordered goods. The order will be assigned to the warehouse for subcontracting of the ordered goods, etc. After the subcontracting is completed, the ordered goods will be assigned to the vehicle for loading, etc. After completion, a transport order will be generated, and the transport will start. After the order is completed, a transport order is generated and transportation begins. After the delivery is completed, the whole order management activity is basically finished.

The inventory management business, which is also an essential business in this system development, is depicted in Figure 4 as an activity diagram. In the logistics management system, warehouse management has always been a key focus, and inventory management and order management operations are inextricably interwoven. The order manager will allocate the order task order to the warehouse manager after the suborder in the order activity. The warehouse administrator will look for the products to be dispatched on the order in the inventory management system and check their stock status based on the information provided. If the goods are not enough or not available, it is necessary to contact the suppliers of the relevant goods for replenishment of goods. When the goods arrive and are warehoused, the administrator needs to carefully register the information of the goods and the warehousing information. In the condition of enough supply, the goods shipping order is generated, and the goods are agreed to leave the warehouse and the information of goods leaving the warehouse is carefully recorded. Subsequently, the goods are be shipped out for subcontracting, subcontracting is completed, and the warehouse administrator will send the shipping task order to the vehicle manager for dispatch. The warehouse management part will also be responsible for the loading of goods and other work to be loaded and out of the warehouse; this time, the warehouse management activities are basically over.

Figure 5 shows the activity diagram of vehicle management; the reasonable scheduling of vehicle management directly determines the efficiency of logistics management, while the vehicle management part is often a relatively large part of the logistics management work overhead. The high cost has been a major problem of the logistics management system; how to control the transportation cost is a major task of the logistics management system; you can start with vehicle transportation management to save costs. In the warehouse for goods out of the warehouse before the generation of transport orders, according to the goods transport orders, vehicle managers will be related to the search work of the vehicle. If there are relevant vehicles that meet the requirements, the generation of the dispatch order will be carried out. If no vehicle meets the requirements, the vehicle will be retrieved from other garages. After the vehicle is retrieved, the loading of goods is carried out, and after the loading is completed, the transportation management of the vehicle is carried out. The vehicle transportation operation is also carried out by the vehicle manager, and the geographic location of the vehicle can be monitored in real time according to the GPS of the vehicle. Until the vehicle is transported, the vehicle administrator is responsible for modifying vehicle information and logistics status information.

### 2.2. System Modeling

According to the above description of the system business process, the use case diagram of the whole system is shown in Figure 6, and the whole system is divided into several different subsystems with the corresponding usage objects of different subsystems. It shows part of the functional modules of the logistics management system and the related participants from a macro perspective. According to the description of the system business logic, the system can be roughly divided into the following modular parts: order management, user management, vehicle management, transportation management, inventory management, data management, and financial management. Different participants can use different functional modules of the system.

The user system is developed based on the B/S model and designed for users. Users can access it through the URL, and if they need to perform business-related operations, such as submitting orders, they need to do so after logging in, but they cannot manage the users, as shown in Figure 7.

The back-office system is developed on a B/S model and is designed for internal managers of logistics companies. After a new order has been placed, the warehouse manager checks the corresponding goods information to ensure that there is a sufficient supply of goods, at the same time, maintains the incoming and outgoing information of the goods in stock, and also adds, deletes, changes, and checks the basic information of the goods and other operations, as shown in Figure 8.

## 3. Implementation of a Logistics Information System

This article describes the implementation of a logistics information system from two aspects, namely, business implementation and technical implementation. Due to space limitations, only the key business and technical implementations are analyzed.

### 3.1. Implementation of the Automatic Order Distribution Business

Following a user's submission of an order in the frontend system, the backend system is contacted remotely to store the order data and do any necessary business logic processing. After receiving order data from the frontend system, the backend system automatically distributes the order based on the information provided and must finally assign an appropriate courier to pick up the products. Two forms of automated order dispatching logic are implemented in the system.

#### 3.1.1. Exact Matching

The exact match from the customer's address is shown in Figure 9. Based on the sender's address in the order information, the customer relationship system is called up remotely. In the customer relationship system, the sender's address is used to find the exact customer in the customer relationship system and when found is returned to the back-office system. This is because in the back-office system, in the zone management, it is possible that in the back-office system, the customer can be linked to a zone in order to match the customer information to the corresponding zone. Finally, the zone is matched to the courier and the backend system calls Ali's larger interface to the courier to send a pickup SMS and generate a courier work order.

#### 3.1.2. Fuzzy Matching

The keyword fuzzy matching according to the partition is shown in Figure 10. In the backend system, based on the provincial and urban area data in the order information, the corresponding regional records are united in the regional table. The corresponding regional records are queried. A region corresponds to multiple partitions, and then the corresponding multiple partition records are then queried. Then, based on the sender's address in the order information to match the address keyword in the partition record, thus the unique partition is determined and then uniquely identified. From the partition to match the unique zone, the final match to the appropriate courier, the backend system calls Alibaba's interface to send a pickup SMS to the courier and generate a courier work order and generates a courier work order.

### 3.2. Message Queues

The implementation of this system involves several remote calls between systems. When a user registers with the frontend system, the user information needs to be passed to the customer relationship system for storage; when logging in, the user information also needs to be passed to the customer relationship system for verification. The order data filled in by the user in the front office system needs to be passed to the back-office system for storage and processing of related operations. This remote call between systems can be implemented using the traditional technology of WebService, but it has the obvious disadvantage that messages cannot be processed asynchronously, only synchronously, and is inefficient. A message queue may be conceived as a container that houses messages that can be taken straight from the container by whoever needs them. Although the logistics information system in this research is not a distributed system, the message queue may be leveraged to enable asynchronous processing for scalable business architecture and enhanced system performance. Message queues can be operated in two different ways: peer-to-peer and publish-subscribe. The message sender, i.e., the producer, publishes a message in the publish-subscribe mode, and multiple message receivers, i.e., consumers, subscribe to the message, as shown in Figure 11.

Figure 11 shows that there is no direct coupling between application A and applications B, C, and D. Once the message queue receives a message from application A, applications B, C, and *D*, which have subscribed to the message, fetch the message from the message queue and process the subsequent operations without the consumer caring about the origin of the message. If you need to add a new service, you can subscribe to the message from the message queue if you are interested in that type of message. This has no impact on the existing system or business, thus enabling the scalability of the site's business design.

As seen in Figure 12, this system exclusively employs the peer-to-peer approach. In other words, a producer transmits a message to only one consumer. For instance, the frontend system sends a message regarding customer registration, but only the customer relationship system receives it, while the backend system does not. In this approach, even if the back-office system is in a maintenance or down state, or even if it is not started, a user who submits an order in the front office system and sends the data to the message queue, the message queue will receive the data. The order data for the backend system will be held in the message queue until the backend system returns to normal. The message queue will then send the data to the backend, even if the backend the message queue will then send the data to the backend, even if the backend system fails to receive it.

Message queues can be used not only for remote calls between systems, but also between the application server and the database server, as shown in Figure 13. The frontend website of a logistics enterprise generates a large amount of order data during peak logistics periods. If these highly concurrent data are written directly to the database, it will put a lot of pressure on the database and even crash. If these highly concurrent data are written directly to the database, it will put a lot of pressure on the database and even crash. The message queue is used to achieve asynchronous processing between the application server and the database. The message queue acts as an asynchronous process between the application server and the database so that the data are not written directly to the database but are first sent to the message queue into the database for immediate return. This allows the data to be written to the database asynchronously. This allows data to be written to the database asynchronously. This allows data to be written to the database asynchronously, resulting in a significant increase in response time for the user and performance for the entire logistics information system.

## 4. Conclusion

With the development of information technology, especially the Internet of Things, and electronic devices, the network platform has just become another area of competition for enterprises in the new era. Only with the combination of emerging computer technology can the traditional industry of logistics once again take on a new life. A more important aspect is the massive data collected through the deployed devices in the closed proximity of the underlined phenomenon. This article takes the current situation of the backward level of information technology in the development of domestic logistics enterprises as the starting point and designs and develops an enterprise logistics information system based on the B/S mode, with the back-office management system as the main system and the front office user system and customer relationship system as the supplementary system. Through this system, the information level of logistics enterprises has been effectively improved, and the management costs of logistics enterprises have been reduced, and a better user experience has been brought to the users. [9–13]

## Figures and Tables

**Figure 1:** The general framework of the B/S-based logistics information system.

**Figure 2:** System business flowchart.

**Figure 3:** Order management activity chart.

**Figure 4:** Inventory management activity chart.

**Figure 5:** Vehicle management activity chart.

**Figure 6:** Logistics information system structure diagram.

**Figure 7:** Order and user business example diagram.

**Figure 8:** Background system based on B/S mode.

**Figure 9:** Order dispatching logic.

**Figure 10:** Keyword fuzzy matching based on partition.

**Figure 11:** Publish-subscribe mode.

**Figure 12:** Peer-to-peer mode.

**Figure 13:** Message queues applied to servers and database servers.

## Data Availability

The datasets used and analyzed during the current study are available from the corresponding author upon reasonable request.
